# Tris[2-(propyl­imino­meth­yl)phenolato-κ^2^ *N*,*O*]iron(III)

This article has been retracted.

**DOI:** 10.1107/S1600536808018540

**Published:** 2008-06-25

**Authors:** Lujiang Hao, Chunhua Mu, Binbin Kong

**Affiliations:** a College of Food and Biological Engineering, Shandong Institute of Light Industry, Jinan 250353, People’s Republic of China; b Maize Research Insitute, Shandong Academy of Agricultural Science, Jinan 250100, People’s Republic of China

## Abstract

The title compound, [Fe(C_10_H_12_NO)_3_], is isostructural with its Co^III^-containing analogue. The Fe^III^ cation is chelated by three Schiff base ligands *via* three N and three O atoms, and exhibits a slightly distorted octa­hedral geometry. The longest Fe—O and Fe—N bonds lie *trans* to each other and may be regarded as axial bonds, while the equatorial plane contains two mutually *trans* O and two *trans* N atoms.

## Related literature

For related literature, see: Iskander *et al.* (2001 ▶); Caruso *et al.* (2005 ▶); Sangeetha & Pal (2000 ▶); Rajak *et al.* (2000 ▶); Sutradhar *et al.* (2006 ▶). For the isostructural Co complex, see: Li *et al.* (2008 ▶).

## Experimental

### 

#### Crystal data

[Fe(C_10_H_12_NO)_3_]
*M* *_r_* = 542.47
Tetragonal,
*a* = 19.369 (2) Å
*c* = 30.216 (3) Å
*V* = 11336 (2) Å^3^
*Z* = 16
Mo *K*α radiation
μ = 0.57 mm^−1^
*T* = 293 (2) K
0.12 × 0.10 × 0.08 mm

#### Data collection

Bruker APEXII CCD diffractometer
Absorption correction: multi-scan (*SADABS*; Bruker, 2001 ▶) *T*_min_ = 0.935, *T*_max_ = 0.956
41740 measured reflections
5198 independent reflections
3125 reflections with *I* > 2σ(*I*)
*R*_int_ = 0.073

#### Refinement

*R*[*F* ^2^ > 2σ(*F* ^2^)] = 0.047
*wR*(*F* ^2^) = 0.099
*S* = 1.00
5198 reflections
337 parameters
H-atom parameters constrained
Δρ_max_ = 0.33 e Å^−3^
Δρ_min_ = −0.27 e Å^−3^

### 

Data collection: *APEX2* (Bruker, 2004 ▶); cell refinement: *SAINT-Plus* (Bruker, 2001 ▶); data reduction: *SAINT-Plus*; program(s) used to solve structure: *SHELXS97* (Sheldrick, 2008 ▶); program(s) used to refine structure: *SHELXL97* (Sheldrick, 2008 ▶); molecular graphics: *SHELXTL* (Sheldrick, 2008 ▶); software used to prepare material for publication: *SHELXTL*.

## Supplementary Material

Crystal structure: contains datablocks global, I. DOI: 10.1107/S1600536808018540/cf2206sup1.cif

Structure factors: contains datablocks I. DOI: 10.1107/S1600536808018540/cf2206Isup2.hkl

Additional supplementary materials:  crystallographic information; 3D view; checkCIF report

## supplementary crystallographic information

### Comment

The design and construction of novel discrete Schiff-basd metal complexes has attracted long-lasting research interest, not only because of their appealing structural and topological features, but also due to their unusual optical, electronic, magnetic and catalytic properties, and their further potential medical value derived from their antiviral properties and inhibition of angiogenesis (Iskander *et al.* 2001; Caruso *et al.* 2005; Sangeetha & Pal, 2000; Rajak *et al.* 2000; Sutradhar *et al.* 2006). Here we report the synthesis and X-ray crystal structure analysis of the title compound, which is isostructural with its Co^III^-containing analogue (Li *et al.*, 2008).

As shown in Figure 1, the Fe^III^ cation is chelated by three Schiff base ligands *via* three N and three O atoms, and exhibits a slightly distorted octahedral geometry. The Fe—N and Fe—O bond lengths are in the ranges 1.917 (3)–1.969 (3) and 1.846 (2)–1.913 (2) Å, respectively. The Fe1—O2 and Fe1—N2 bonds are much longer than the other related ones. Thus the atoms O1, O3, N1, and N3 may be considered to lie in the equatorial plane, and O2 and N2 in the axial coordination sites.

### Experimental

A mixture of iron(III) acetylacetonate (0.5 mmol) and 2-(propyliminomethyl)phenol (0.5 mmol) in 20 ml methanol was refluxed for several hours. The filtrate obtained from this soution was allowed to evaporate at room temperature for three days. Brown crystals were obtained with a yield of 5%. Anal. Calc. for C_30_H_36_FeN_3_O_3_: C 65.36, H 6.64 N 7.74%; Found: C 65.21, H 6.59, N 7.67%.

### Refinement

All H atoms were placed in calculated positions with C—H = 0.93Å and refined as riding with *U*_iso_(H) = 1.2*U*_eq_(C).

### Crystal data

**Table:**

[Fe(C_10_H_12_N_1_O_1_)_3_]	*Z* = 16
*M**_r_* = 542.47	*F*_000_ = 4592
Tetragonal, *I*4_1_/*a*	*D*_x_ = 1.271 Mg m^−^^3^
Hall symbol: -I 4ad	Mo *K*α radiation λ = 0.71073 Å
*a* = 19.369 (2) Å	Cell parameters from 5198 reflections
*b* = 19.369 (2) Å	θ = 1.3–25.5º
*c* = 30.216 (3) Å	µ = 0.57 mm^−^^1^
α = 90º	*T* = 293 (2) K
β = 90º	Block, green
γ = 90º	0.12 × 0.10 × 0.08 mm
*V* = 11336 (2) Å^3^	

### Data collection

**Table:**

Bruker APEXII CCD diffractometer	5198 independent reflections
Radiation source: fine-focus sealed tube	3125 reflections with *I* > 2σ(*I*)
Monochromator: graphite	*R*_int_ = 0.073
*T* = 293(2) K	θ_max_ = 25.5º
φ and ω scans	θ_min_ = 1.3º
Absorption correction: multi-scan(SADABS; Bruker, 2001)	*h* = −23→22
*T*_min_ = 0.935, *T*_max_ = 0.956	*k* = −23→23
41740 measured reflections	*l* = −36→36

### Refinement

**Table:**

Refinement on *F*^2^	Secondary atom site location: difference Fourier map
Least-squares matrix: full	Hydrogen site location: inferred from neighbouring sites
*R*[*F*^2^ > 2σ(*F*^2^)] = 0.047	H-atom parameters constrained
*wR*(*F*^2^) = 0.099	*w* = 1/[σ^2^(*F*_o_^2^) + (0.0375*P*)^2^] where *P* = (*F*_o_^2^ + 2*F*_c_^2^)/3
*S* = 1.00	(Δ/σ)_max_ < 0.001
5198 reflections	Δρ_max_ = 0.33 e Å^−^^3^
337 parameters	Δρ_min_ = −0.27 e Å^−^^3^
Primary atom site location: structure-invariant direct methods	Extinction correction: none

### Special details

**Table:**

Geometry. All e.s.d.'s (except the e.s.d. in the dihedral angle between two l.s. planes) are estimated using the full covariance matrix. The cell e.s.d.'s are taken into account individually in the estimation of e.s.d.'s in distances, angles and torsion angles; correlations between e.s.d.'s in cell parameters are only used when they are defined by crystal symmetry. An approximate (isotropic) treatment of cell e.s.d.'s is used for estimating e.s.d.'s involving l.s. planes.
Refinement. Refinement of *F*^2^ against ALL reflections. The weighted *R*-factor *wR* and goodness of fit *S* are based on *F*^2^, conventional *R*-factors *R* are based on *F*, with *F* set to zero for negative *F*^2^. The threshold expression of *F*^2^ > σ(*F*^2^) is used only for calculating *R*-factors(gt) *etc*. and is not relevant to the choice of reflections for refinement. *R*-factors based on *F*^2^ are statistically about twice as large as those based on *F*, and *R*- factors based on ALL data will be even larger.

### Fractional atomic coordinates and isotropic or equivalent isotropic displacement parameters (Å^2^)

**Table:**

	*x*	*y*	*z*	*U*_iso_*/*U*_eq_	
Fe1	0.22632 (2)	0.98149 (2)	0.992992 (13)	0.05735 (17)	
C1	0.14742 (16)	0.94922 (15)	0.89961 (9)	0.0579 (8)	
C2	0.10654 (19)	0.94259 (17)	0.86092 (10)	0.0703 (9)	
H2	0.1202	0.9650	0.8352	0.084*	
C3	0.04851 (19)	0.90467 (18)	0.86056 (12)	0.0783 (10)	
H3	0.0213	0.9020	0.8353	0.094*	
C4	0.03008 (16)	0.86948 (17)	0.89893 (12)	0.0755 (9)	
H4	−0.0097	0.8426	0.8989	0.091*	
C5	0.06917 (16)	0.87330 (15)	0.93694 (10)	0.0647 (8)	
H5	0.0554	0.8488	0.9619	0.078*	
C6	0.12904 (15)	0.91330 (14)	0.93872 (10)	0.0548 (7)	
C7	0.09561 (16)	0.97163 (15)	1.05726 (9)	0.0577 (8)	
C8	0.03352 (16)	0.95695 (16)	1.07764 (10)	0.0693 (9)	
H8	−0.0047	0.9843	1.0713	0.083*	
C9	0.02656 (19)	0.90334 (17)	1.10688 (11)	0.0745 (9)	
H9	−0.0158	0.8943	1.1202	0.089*	
C10	0.0822 (2)	0.86399 (18)	1.11603 (10)	0.0749 (9)	
H10	0.0774	0.8266	1.1351	0.090*	
C11	0.14583 (19)	0.87783 (16)	1.09771 (10)	0.0706 (9)	
H11	0.1836	0.8506	1.1053	0.085*	
C12	0.15458 (16)	0.93302 (15)	1.06737 (9)	0.0561 (8)	
C13	0.34061 (18)	1.0494 (2)	1.03341 (11)	0.0738 (9)	
C14	0.3673 (2)	1.1078 (2)	1.05590 (13)	0.1009 (12)	
H14	0.3404	1.1474	1.0587	0.121*	
C15	0.4327 (2)	1.1063 (3)	1.07356 (14)	0.1233 (17)	
H15	0.4494	1.1449	1.0885	0.148*	
C16	0.4732 (2)	1.0498 (3)	1.06961 (15)	0.1199 (16)	
H16	0.5172	1.0495	1.0819	0.144*	
C17	0.4490 (2)	0.9930 (3)	1.04737 (13)	0.1051 (13)	
H17	0.4772	0.9544	1.0445	0.126*	
C18	0.38262 (17)	0.9922 (2)	1.02892 (11)	0.0764 (10)	
C19	0.36133 (19)	0.9318 (2)	1.00561 (11)	0.0781 (10)	
H19	0.3945	0.8974	1.0026	0.094*	
C20	0.20828 (17)	0.98920 (16)	0.89763 (11)	0.0678 (9)	
H20	0.2235	1.0028	0.8698	0.081*	
C21	0.09974 (16)	1.02899 (16)	1.02768 (10)	0.0660 (8)	
H21	0.0631	1.0600	1.0285	0.079*	
C22	0.14568 (17)	1.10734 (17)	0.97424 (12)	0.0844 (10)	
H22A	0.1397	1.0951	0.9433	0.101*	
H22B	0.1903	1.1297	0.9769	0.101*	
C23	0.0919 (2)	1.15896 (17)	0.98566 (12)	0.0889 (11)	
H23A	0.0971	1.1730	1.0163	0.107*	
H23B	0.0465	1.1386	0.9821	0.107*	
C24	0.0987 (2)	1.22091 (17)	0.95597 (13)	0.1048 (13)	
H24A	0.1464	1.2340	0.9539	0.157*	
H24B	0.0725	1.2586	0.9680	0.157*	
H24C	0.0814	1.2098	0.9270	0.157*	
C25	0.3097 (2)	1.0451 (3)	0.92058 (14)	0.1238 (15)	
H25A	0.3341	1.0515	0.9483	0.149*	
H25B	0.3373	1.0136	0.9029	0.149*	
C26	0.3106 (3)	1.1023 (3)	0.9010 (2)	0.126 (3)	
H26A	0.2831	1.1346	0.9182	0.240*	
H26B	0.2878	1.0966	0.8727	0.240*	
C27	0.3813 (2)	1.1356 (2)	0.89256 (15)	0.1331 (17)	
H27A	0.3935	1.1643	0.9173	0.200*	
H27B	0.3792	1.1632	0.8662	0.200*	
H27C	0.4154	1.1001	0.8890	0.200*	
C28	0.29461 (18)	0.85217 (19)	0.96588 (12)	0.0870 (11)	
H28A	0.3396	0.8358	0.9565	0.104*	
H28B	0.2665	0.8584	0.9396	0.104*	
C29	0.2615 (2)	0.7984 (2)	0.99533 (14)	0.1041 (13)	
H29A	0.2164	0.8152	1.0043	0.125*	
H29B	0.2541	0.7569	0.9779	0.125*	
C30	0.3005 (2)	0.7793 (2)	1.03570 (18)	0.1528 (19)	
H30A	0.3439	0.7591	1.0274	0.229*	
H30B	0.2743	0.7465	1.0526	0.229*	
H30C	0.3087	0.8198	1.0532	0.229*	
N1	0.30265 (14)	0.91895 (14)	0.98831 (8)	0.0679 (7)	
N2	0.24462 (14)	1.00853 (13)	0.93127 (9)	0.0697 (7)	
N3	0.14842 (12)	1.04268 (13)	0.99995 (8)	0.0635 (7)	
O1	0.27883 (11)	1.05426 (11)	1.01689 (7)	0.0753 (6)	
O2	0.21526 (10)	0.94675 (11)	1.05183 (6)	0.0651 (6)	
O3	0.16501 (10)	0.91380 (10)	0.97551 (6)	0.0622 (5)	

### Atomic displacement parameters (Å^2^)

**Table:**

	*U*^11^	*U*^22^	*U*^33^	*U*^12^	*U*^13^	*U*^23^
Fe1	0.0520 (3)	0.0673 (3)	0.0527 (3)	0.0034 (2)	0.0019 (2)	−0.0006 (2)
C1	0.068 (2)	0.0595 (19)	0.0458 (18)	0.0098 (17)	0.0056 (16)	−0.0015 (15)
C2	0.092 (3)	0.071 (2)	0.049 (2)	0.010 (2)	0.0032 (18)	−0.0026 (16)
C3	0.086 (3)	0.086 (3)	0.063 (2)	0.001 (2)	−0.011 (2)	−0.0124 (19)
C4	0.064 (2)	0.079 (2)	0.084 (3)	0.0000 (18)	−0.007 (2)	−0.021 (2)
C5	0.066 (2)	0.062 (2)	0.066 (2)	0.0029 (17)	0.0066 (17)	−0.0042 (16)
C6	0.060 (2)	0.0522 (18)	0.0517 (19)	0.0087 (15)	0.0042 (16)	−0.0050 (15)
C7	0.064 (2)	0.0522 (18)	0.0571 (19)	0.0062 (16)	0.0055 (16)	−0.0028 (15)
C8	0.070 (2)	0.064 (2)	0.074 (2)	0.0055 (17)	0.0133 (18)	−0.0013 (18)
C9	0.085 (3)	0.068 (2)	0.070 (2)	−0.005 (2)	0.0171 (19)	−0.0010 (19)
C10	0.104 (3)	0.064 (2)	0.057 (2)	−0.006 (2)	0.013 (2)	0.0015 (16)
C11	0.095 (3)	0.062 (2)	0.055 (2)	0.0135 (19)	−0.0056 (19)	−0.0051 (17)
C12	0.067 (2)	0.0582 (19)	0.0436 (17)	0.0072 (17)	0.0007 (16)	−0.0091 (15)
C13	0.057 (2)	0.095 (3)	0.069 (2)	−0.010 (2)	0.0062 (18)	−0.006 (2)
C14	0.072 (3)	0.126 (3)	0.105 (3)	−0.012 (2)	0.004 (2)	−0.034 (3)
C15	0.074 (3)	0.184 (5)	0.112 (3)	−0.033 (3)	−0.001 (3)	−0.050 (3)
C16	0.065 (3)	0.183 (5)	0.112 (4)	−0.007 (3)	−0.016 (3)	−0.023 (4)
C17	0.061 (3)	0.153 (4)	0.101 (3)	0.001 (3)	0.000 (2)	−0.001 (3)
C18	0.053 (2)	0.106 (3)	0.070 (2)	0.004 (2)	0.0030 (18)	−0.002 (2)
C19	0.066 (2)	0.095 (3)	0.074 (2)	0.019 (2)	0.013 (2)	0.002 (2)
C20	0.074 (2)	0.077 (2)	0.052 (2)	0.0004 (19)	0.0096 (17)	0.0060 (17)
C21	0.060 (2)	0.064 (2)	0.074 (2)	0.0074 (17)	0.0052 (17)	0.0079 (17)
C22	0.075 (2)	0.079 (2)	0.099 (3)	0.005 (2)	0.015 (2)	0.027 (2)
C23	0.104 (3)	0.074 (2)	0.089 (3)	0.007 (2)	−0.005 (2)	0.002 (2)
C24	0.130 (3)	0.065 (2)	0.120 (3)	0.001 (2)	−0.008 (3)	0.021 (2)
C25	0.127 (4)	0.144 (4)	0.100 (3)	−0.035 (3)	−0.002 (3)	0.037 (3)
C26	0.148 (8)	0.122 (7)	0.110 (7)	−0.007 (6)	−0.014 (6)	−0.005 (6)
C27	0.124 (4)	0.118 (3)	0.157 (4)	−0.063 (3)	0.028 (3)	0.000 (3)
C28	0.080 (3)	0.092 (3)	0.089 (3)	0.021 (2)	0.007 (2)	−0.024 (2)
C29	0.108 (3)	0.076 (3)	0.129 (4)	0.014 (2)	0.000 (3)	0.007 (3)
C30	0.139 (4)	0.138 (4)	0.182 (5)	0.003 (3)	−0.040 (4)	0.040 (4)
N1	0.0608 (17)	0.083 (2)	0.0596 (16)	0.0104 (15)	0.0072 (14)	−0.0056 (14)
N2	0.0630 (17)	0.0785 (19)	0.0675 (18)	−0.0054 (15)	0.0064 (15)	0.0089 (15)
N3	0.0560 (15)	0.0691 (17)	0.0653 (17)	0.0024 (13)	0.0007 (13)	0.0120 (14)
O1	0.0568 (14)	0.0766 (15)	0.0925 (17)	0.0006 (12)	−0.0033 (12)	−0.0077 (12)
O2	0.0572 (13)	0.0848 (15)	0.0532 (12)	0.0147 (11)	−0.0012 (10)	−0.0047 (11)
O3	0.0650 (13)	0.0710 (14)	0.0506 (12)	−0.0013 (10)	−0.0026 (10)	0.0063 (10)

### Geometric parameters (Å, °)

**Table:**

Fe1—O3	1.846 (2)	C17—C18	1.402 (5)
Fe1—O1	1.882 (2)	C17—H17	0.930
Fe1—O2	1.913 (2)	C18—C19	1.425 (5)
Fe1—N1	1.917 (3)	C19—N1	1.276 (4)
Fe1—N3	1.930 (2)	C19—H19	0.930
Fe1—N2	1.969 (3)	C20—N2	1.292 (4)
C1—C20	1.412 (4)	C20—H20	0.930
C1—C2	1.418 (4)	C21—N3	1.289 (3)
C1—C6	1.417 (4)	C21—H21	0.930
C2—C3	1.343 (4)	C22—N3	1.475 (4)
C2—H2	0.930	C22—C23	1.484 (4)
C3—C4	1.392 (4)	C22—H22A	0.970
C3—H3	0.930	C22—H22B	0.970
C4—C5	1.378 (4)	C23—C24	1.504 (4)
C4—H4	0.930	C23—H23A	0.970
C5—C6	1.396 (4)	C23—H23B	0.970
C5—H5	0.930	C24—H24A	0.960
C6—O3	1.312 (3)	C24—H24B	0.960
C7—C8	1.381 (4)	C24—H24C	0.960
C7—C12	1.399 (4)	C25—C26	1.257 (5)
C7—C21	1.428 (4)	C25—N2	1.481 (5)
C8—C9	1.370 (4)	C25—H25A	0.970
C8—H8	0.930	C25—H25B	0.970
C9—C10	1.348 (4)	C26—C27	1.535 (6)
C9—H9	0.930	C26—H26A	0.970
C10—C11	1.378 (4)	C26—H26B	0.970
C10—H10	0.930	C27—H27A	0.960
C11—C12	1.418 (4)	C27—H27B	0.960
C11—H11	0.930	C27—H27C	0.960
C12—O2	1.293 (3)	C28—N1	1.469 (4)
C13—O1	1.300 (4)	C28—C29	1.514 (5)
C13—C18	1.382 (5)	C28—H28A	0.970
C13—C14	1.418 (5)	C28—H28B	0.970
C14—C15	1.376 (5)	C29—C30	1.482 (5)
C14—H14	0.930	C29—H29A	0.970
C15—C16	1.352 (6)	C29—H29B	0.970
C15—H15	0.930	C30—H30A	0.960
C16—C17	1.372 (5)	C30—H30B	0.960
C16—H16	0.930	C30—H30C	0.960
			
O3—Fe1—O1	171.58 (9)	N2—C20—C1	125.5 (3)
O3—Fe1—O2	86.80 (8)	N2—C20—H20	117.2
O1—Fe1—O2	88.13 (9)	C1—C20—H20	117.2
O3—Fe1—N1	91.50 (11)	N3—C21—C7	127.4 (3)
O1—Fe1—N1	94.86 (11)	N3—C21—H21	116.3
O2—Fe1—N1	86.14 (9)	C7—C21—H21	116.3
O3—Fe1—N3	87.97 (10)	N3—C22—C23	118.4 (3)
O1—Fe1—N3	85.46 (10)	N3—C22—H22A	107.7
O2—Fe1—N3	91.56 (9)	C23—C22—H22A	107.7
N1—Fe1—N3	177.67 (10)	N3—C22—H22B	107.7
O3—Fe1—N2	91.93 (10)	C23—C22—H22B	107.7
O1—Fe1—N2	93.83 (11)	H22A—C22—H22B	107.1
O2—Fe1—N2	173.65 (9)	C22—C23—C24	109.7 (3)
N1—Fe1—N2	87.67 (10)	C22—C23—H23A	109.7
N3—Fe1—N2	94.62 (10)	C24—C23—H23A	109.7
C20—C1—C2	118.8 (3)	C22—C23—H23B	109.7
C20—C1—C6	121.0 (3)	C24—C23—H23B	109.7
C2—C1—C6	120.2 (3)	H23A—C23—H23B	108.2
C3—C2—C1	121.6 (3)	C23—C24—H24A	109.5
C3—C2—H2	119.2	C23—C24—H24B	109.5
C1—C2—H2	119.2	H24A—C24—H24B	109.5
C2—C3—C4	118.4 (3)	C23—C24—H24C	109.5
C2—C3—H3	120.8	H24A—C24—H24C	109.5
C4—C3—H3	120.8	H24B—C24—H24C	109.5
C5—C4—C3	121.8 (3)	C26—C25—N2	122.4 (5)
C5—C4—H4	119.1	C26—C25—H25A	106.7
C3—C4—H4	119.1	N2—C25—H25A	106.7
C4—C5—C6	121.2 (3)	C26—C25—H25B	106.7
C4—C5—H5	119.4	N2—C25—H25B	106.7
C6—C5—H5	119.4	H25A—C25—H25B	106.6
O3—C6—C5	118.6 (3)	C25—C26—C27	117.4 (5)
O3—C6—C1	124.7 (3)	C25—C26—H26A	108.0
C5—C6—C1	116.7 (3)	C27—C26—H26A	107.9
C8—C7—C12	120.2 (3)	C25—C26—H26B	107.9
C8—C7—C21	119.2 (3)	C27—C26—H26B	107.9
C12—C7—C21	120.5 (3)	H26A—C26—H26B	107.2
C9—C8—C7	122.0 (3)	C26—C27—H27A	109.5
C9—C8—H8	119.0	C26—C27—H27B	109.5
C7—C8—H8	119.0	H27A—C27—H27B	109.5
C10—C9—C8	118.8 (3)	C26—C27—H27C	109.5
C10—C9—H9	120.6	H27A—C27—H27C	109.5
C8—C9—H9	120.6	H27B—C27—H27C	109.5
C9—C10—C11	121.5 (3)	N1—C28—C29	112.3 (3)
C9—C10—H10	119.2	N1—C28—H28A	109.1
C11—C10—H10	119.2	C29—C28—H28A	109.1
C10—C11—C12	120.9 (3)	N1—C28—H28B	109.1
C10—C11—H11	119.6	C29—C28—H28B	109.1
C12—C11—H11	119.6	H28A—C28—H28B	107.9
O2—C12—C7	123.5 (3)	C30—C29—C28	116.0 (4)
O2—C12—C11	119.9 (3)	C30—C29—H29A	108.3
C7—C12—C11	116.5 (3)	C28—C29—H29A	108.3
O1—C13—C18	124.2 (3)	C30—C29—H29B	108.3
O1—C13—C14	117.5 (4)	C28—C29—H29B	108.3
C18—C13—C14	118.3 (3)	H29A—C29—H29B	107.4
C15—C14—C13	120.3 (4)	C29—C30—H30A	109.5
C15—C14—H14	119.9	C29—C30—H30B	109.5
C13—C14—H14	119.9	H30A—C30—H30B	109.5
C14—C15—C16	121.2 (4)	C29—C30—H30C	109.5
C14—C15—H15	119.4	H30A—C30—H30C	109.5
C16—C15—H15	119.4	H30B—C30—H30C	109.5
C15—C16—C17	119.6 (4)	C19—N1—C28	117.1 (3)
C15—C16—H16	120.2	C19—N1—Fe1	122.2 (2)
C17—C16—H16	120.2	C28—N1—Fe1	120.6 (2)
C16—C17—C18	121.2 (4)	C20—N2—C25	115.5 (3)
C16—C17—H17	119.4	C20—N2—Fe1	124.7 (2)
C18—C17—H17	119.4	C25—N2—Fe1	119.1 (2)
C17—C18—C13	119.5 (4)	C21—N3—C22	119.4 (3)
C17—C18—C19	118.1 (4)	C21—N3—Fe1	121.1 (2)
C13—C18—C19	122.4 (3)	C22—N3—Fe1	119.5 (2)
N1—C19—C18	128.3 (3)	C13—O1—Fe1	126.2 (2)
N1—C19—H19	115.8	C12—O2—Fe1	120.76 (18)
C18—C19—H19	115.8	C6—O3—Fe1	126.11 (18)
